# Diagnostic Accuracy of Salivary Biomarkers including Lactate Dehydrogenase and Hemoglobin A1c for Screening Chronic Periodontitis

**DOI:** 10.1155/2022/1119038

**Published:** 2022-04-26

**Authors:** Somaye Ansari Moghadam, Fateme Soude Ahmadi Moghadam, Ebrahim Alijani

**Affiliations:** ^1^Associate Professor, Department of Periodontology, Oral and Dental Disease Research Center, Zahedan University of Medical Sciences, Zahedan, Iran; ^2^Dentist, Oral and Dental Disease Research Center, Zahedan University of Medical Sciences, Zahedan, Iran; ^3^Department of Clinical Immunology Research Center, Zahedan University of Medical Sciences, Zahedan, Iran

## Abstract

*Aims*: Periodontitis is one of the most common chronic bacterial infections in humans involving the tooth-supporting tissue. The present study aimed to evaluate and compare salivary biomarkers, including lactate dehydrogenase (LDH) and hemoglobin A1c (HbA1c), between patients with severe chronic periodontitis and healthy individuals. *Methods*: This study was performed on 29 patients with severe chronic periodontitis and 30 healthy individuals at Zahedan University of Medical Sciences, Zahedan, Iran, in 2021. Salivary samples were taken, and clinical parameters, including the clinical attachment loss (CAL) and probing pocket depth (PPD), were measured. Besides, the levels of LDH and HbA1c were measured using ELISA kits. The sensitivity, specificity, and positive and negative predictive values of HbA1c and LDH were examined for chronic periodontitis diagnosis. *Results*: Based on the present results, the levels of LDH and HbA1C did not show adequate sensitivity or specificity for screening chronic periodontitis. *Conclusion*: According to the present findings, salivary biomarkers, including LDH and HbA1c, cannot be used with certainty for screening chronic periodontitis.

## 1. Introduction

Periodontitis is one of the most common chronic bacterial infections in humans, involving the tooth-supporting tissue. It is recognized as one of the main causes of tooth loss in adults [1]. This disease has two distinct, but interrelated components, including bacteria and the host inflammatory mediators. Periodontal pathogens directly induce the production of biologically active molecules affecting the host tissue and stimulate the production of host inflammatory mediators, leading to tissue and bone destruction [2].

Conventional screening methods for periodontitis include measurement of the probing pocket depth (PPD) by a dentist. The community periodontal index (CPI) is also a scoring system for screening periodontal disease. Besides, saliva has been suggested as an important biological fluid for diagnosis and explanation of the pathogenesis of some systemic diseases. Overall, the host response to periodontal disease involves the production of various enzymes, released due to damage and death of stromal, epithelial, or inflammatory cells [3, 4]. Different salivary biomarkers have been evaluated yet.

In this regard, a study by Hamodat et al. (2019), evaluating the salivary levels of tumor necrosis factor-*α* (TNF-*α*) and LDH, reported no significant difference in the mean serum TNF-*α* concentration between patients with chronic periodontitis and healthy controls. On the other hand, the mean LDH level was significantly higher in the patients compared to the controls; however, there was no significant relationship between the salivary level of LDH and clinical attachment loss (CAL) or PPD [5].

Moreover, Sabarathinam et al. (2019) examined the salivary Hb level and investigated its efficacy in periodontal disease screening. Their results showed that the mean level of salivary Hb was significantly higher in the periodontitis and gingivitis groups compared to the controls. It seems that salivary hemoglobin levels can be used as a non-invasive and economic tool for periodontal screening [6]. Also, Miyoshi et al. (2018) performed a study in Japan on the relationship between salivary LDH levels and systemic inflammation. Their results showed that salivary LDH had a strong positive correlation with the periodontal status, as higher levels of LDH were associated with higher levels of systemic inflammatory markers [7].

Additionally, Moradi Haghgoo et al. (2016) compared the LDH levels of patients with periodontitis and healthy individuals, referred to Hamadan Dental School, Hamadan, Iran. Their findings showed that the mean LDH level in the periodontitis group was significantly higher than that of the control group (P <0.05) [8]. Besides, Maeng et al. (2016), in a study in South Korea, examined the diagnostic accuracy of salivary Hb levels for periodontitis screening. Their results indicated that salivary Hb was significantly higher in patients with periodontitis; however, no positive correlation was found between the periodontal index and Hb level [9].

Another study by Nomura et al. (2016) in Japan investigated the diagnostic validity of salivary biomarkers, including LDH and Hb, as new tools for screening periodontitis and suitable alternatives to the periodontal index. Their results showed that LDH and Hb levels were significantly higher in patients with periodontitis compared to the healthy individuals. However, there was no significant correlation between the periodontal index and salivary LDH and Hb levels in either of the groups [10]. Kugahara et al. (2008) also performed a study in Japan on periodontitis screening in pregnant women, based on salivary enzymes. They determined the salivary enzyme levels to evaluate the periodontitis status before dental examinations. Their results showed that LDH and alkaline phosphatase (ALP) levels were significantly higher in patients with periodontitis compared to those with gingivitis and healthy individuals [11].

A study by De La Peña et al. (2007), entitled “Relationship between lactate dehydrogenase activity in saliva and oral health status”, showed that LDH was positively correlated with the periodontal index; in other words, a PPD above 5 mm indicated a higher LDH level. It seems that salivary LDH level can be a reliable biomarker for the periodontal status [12]. In this regard, a study by Nomura et al. (2006) in Japan on periodontitis screening using salivary enzymes showed that LDH and Hb levels were significantly higher in patients with periodontal disease (gingivitis and periodontitis) compared to healthy individuals. Also, the level of these markers increased with the exacerbation of periodontal disease, showing a significant positive correlation between these biomarkers and the periodontal index [13].

Another study by Ruchika et al. (2012) in India compared the HbA1c levels between patients with non-diabetic periodontitis and healthy individuals. Their findings showed that HbA1c level was higher in patients than in healthy individuals; however, the difference was non-significant between the two groups [14]. On the other hand, a study by Ansari et al. (2014) revealed that HbA1c was higher in non-diabetic healthy individuals compared to their counterparts without chronic periodontitis [15].

Study by Isola showed that, Non-Like receptor Family Pyrin domain containing protein 3(NLRP3), plays an important role in the development of periodontitis and diabetes. The presence of periodontitis was a strong predictor of increased NLRP3 ‘s serum and salivary concentrations [16].

Ferlazzo ‘s study found that hypermethylation of cancer related genes, even oral cancers, may be affected by polymorphism of Methylene tetrahydro folate reductase (MTHER) [17].

Conventional periodontal screening methods, is maybe painful and time consuming for patients specially pregnant women, but salivary biomarkers measuring, has been suggested as an important fluid for diagnosis of some systemic disease. Salivary lactate dehydrogenase (LDH) and hemoglobin (Hb) levels are new biomarkers for screening periodontal disease. Measurement of these biomarkers is generally easier than CPI, especially in pregnant women for periodontitis screening. Glycosylated hemoglobin A1c (HbA1c) is a form of hemoglobin, which is mainly used to measure the average blood glucose levels. The HbA1c test measures the average blood glucose over the last two or three months. It particularly reflects the percentage of hemoglobin, a protein bound to glucose. The target HbA1c level is below 7% in the treatment of patients with diabetes. Many studies have reported a significant relationship between the HbA1C level and pregnancy complications [4]. Given the contradictions between the results of Ansari Moghadam's study [15] and other previous studies regarding the diagnostic validity of HbA1C in periodontitis and diabetes, the present study aimed to assess the value of HbA1C as a one of biomarkers.

It should be noted that measurement of free Hb (FHb) and LDH was preferable in this study; however, owing to the high cost and unavailability of the FHb kit in Iran (due to sanctions), the HbA1C biomarker was examined inevitably.

## 2. Material and Methods

This study aimed to determine the diagnostic accuracy of salivary biomarkers, including LDH and HbA1c, for periodontal disease screening in Zahedan Faculty of Dentistry, Zahedan, Iran. Patients with chronic periodontitis, presenting to the Department of Periodontics of Zahedan Faculty of Dentistry, were included in the study after obtaining informed consent. The patients' companions were enrolled as healthy individuals.

The inclusion criteria for group A (control group) were as follows: individuals with oral systemic health; normal body mass index (BMI) of 18-25 kg/m^2^; lack of PDD ≥3; CAL; use of antibiotics or periodontal treatment within the last six months; use of tobacco or drugs affecting the saliva; pregnancy or lactation; and diabetes [16]. The subjects' teeth were plaque-free clinically with no signs of gingivitis. Some subjects had <10% dental plaques (dental plaques were found in all subjects), but did not require advanced periodontal treatment. Moreover, the inclusion criteria for group B (chronic periodontitis group) were as follows: individuals with oral systemic health; BMI of 18-25 kg/m^2^; CAL ≥5 in at least two teeth; lack of tobacco use; use of drugs or antibiotics affecting the saliva or periodontal disease medications within the last six months; lack of pregnancy or lactation; and lack of diabetes [18].

Periodontal examinations were performed after collecting the demographic information and intraoral examinations for pathological problems. All examinations were performed by one professional person to remove bias effect. Before collecting salivary samples, the study objectives and procedures were explained to the participants, and written consent was obtained from all of them. The subjects were asked to abstain from eating or drinking for at least two hours before collecting the saliva. They also rinsed their mouth with water for one minute before collecting the salivary samples.

Next, spit it into sterile 15-mL Falcon tubes. A 3-mL salivary sample was taken from all participants. The tubes were temporarily stored at -20°C and then sent to the immunology laboratory to be stored at -70°C until further testing. After sampling, salivary parameters, including HbA1c and LDH, were examined using ELISA kits, according to the manufacturer's instructions (Hangzhou East Biopharm Co., Ltd.CHINA).

Data analysis.

Data were entered into SPSS version 25. The sensitivity, specificity, and positive and negative predictive values were measured to represent the data.

## 3. Results

In the present study, 29 patients with periodontitis and 30 healthy individuals were enrolled. In the patient group, 37.9% were male, and 62.1% were female; also, in the control group, 40% were male, and 60% were female. The results of Fisher's exact test showed a similar gender distribution in the two groups. The mean age of the patient and control groups was 37.85 ± 10.78 and 35.93 ± 10.58 years, respectively; the two groups were matched in terms of age, based on the *P*-value.

The results presented in Table 1 show no significant differences in the HbA1c and LDH levels between subjects with the CPI scores of 0, 3, and 4. The PDD was similar for patients with CPI scores of 3 and 4, whereas the CAL score was significantly higher in subjects with a CPI score of 4 versus those with a CPI score of 3 (P <0.001).

The results presented in Table 2 show that the HbA1c level was significantly lower in patients with periodontitis as compared to the healthy individuals; however, the LDH levels were higher in the periodontitis group compared to the healthy individuals, although the difference was not statistically significant.

Moreover, the ROC curve analysis was performed to evaluate the diagnostic value of salivary HbA1c and LDH levels for periodontitis. The area under the ROC curve (AUC) for salivary HbA1c was 0.38 (95% confidence level [CI]: 0.2358-0.538). The cutoff point of 257 showed the optimal balance of sensitivity and specificity (64% vs. 27%), with positive and negative predictive values of 51% and 27%, respectively. The low sensitivity, specificity, and positive and predictive values indicated the low diagnostic value of this biomarker. The AUC also indicated the low diagnostic value of salivary HbA1c for periodontitis (Table 3).

Regarding salivary LDH, the AUC was measured to be 0.58 (95% CI: 0.412-0.762). The cutoff point of 272 showed the optimal balance of sensitivity and specificity (50% vs. 46%), with positive and negative predictive values of 20% and 76%, respectively. The low sensitivity, specificity, and positive and negative predictive values suggested the low diagnostic value of the tested method. The AUC also revealed the low diagnostic value of salivary LDH for periodontitis. Overall, the positive predictive value was higher for salivary HbA1c than LDH. A positive predictive value of 51% for HbA1c suggested that salivary HbA1c corresponded to the clinical findings by 51%, while salivary LDH was consistent with 20% of the clinical results (Figures 1–2).

## 4. Discussion

The present results showed a significant relationship between the HbA1c level and chronic periodontitis. In contrast to our findings, Ruchika et al. reported an insignificant relationship between the HbA1c level and chronic periodontitis [14], while Hideaki et al. [19] and Padma et al. [20] found a significant correlation between HbA1c level and chronic periodontitis. In contrast to studies which reported higher HbA1c levels in patients with periodontitis compared to healthy individuals, the HbA1c levels were higher in the healthy controls in our study compared to those with chronic periodontitis. These results are in line with the findings reported by Ansari et al. (2014) [15]. Owing to discrepancy between the results, HbA1c may not be a reliable diagnostic marker for examining the risk of diabetes in non-diabetic patients with chronic periodontitis.

The present findings are consistent with those of a study by Pajunen et al. [21] which reported the low sensitivity of HbA1c for diabetes diagnosis; overall, 61% of patients with diabetes had HbA1c <6.5%, and HbA1c assessment delayed the diagnosis of diabetes in 61% of the patients. Lorenzo et al. [22] also reported that HbA1c might not be applicable for diagnosing diabetes; it could be only used to monitor diabetes progression. Similarly, Sonia SA et al. [23] did not consider HbA1c to be a reliable marker for diabetes diagnosis, because it is influenced by factors, such as malaria, anemia, race, and infection, which may partly justify the contradictions between the present and previous findings.

Another shortcoming of the HbA1c test is the inaccuracy of measurements and lack of standardization [5]. In the present study, the AUC for HbA1C was 0.38. The cutoff point of 257 also showed the optimal balance of sensitivity and specificity (64% vs. 27%), with positive and negative predictive values of 51% and 27%, respectively. Overall, the low sensitivity, specificity, and positive and negative predictive values indicated the low diagnostic value of this biomarker. Also, the AUC indicated the low diagnostic value of HbA1C for periodontitis.

Various studies have reported higher levels of LDH in periodontitis patients compared to healthy individuals [4, 5]. The results of a study by Miyoshi et al. (2018) also showed that the serum LDH level is a strong indicator of the periodontal status. The serum LDH was significantly correlated with inflammatory and systemic markers and consequently, the disease. Therefore, systemic diseases may be regarded as confounding factors in LDH measurements [7]. Although these results are consistent with the present findings, the association was insignificant in our study.

In the present study, the AUC for salivary LDH was 0.58. The cutoff point of 272 also showed the optimal balance of sensitivity and specificity (46% vs. 50%), with positive and negative predictive values of 20% and 76%, respectively. The low sensitivity, specificity, and positive and negative predictive values suggested the low diagnostic value of the tested method. The AUC also revealed the low diagnostic value of salivary LDH for periodontitis.

In a study by Nomura et al. (2016) on a new screening method for periodontitis using salivary biomarkers, including LDH and HbA1c as alternatives to the periodontal index, no significant correlation was found between the periodontal index and salivary LDH [10]; these findings are in line with those of the present study. However, the study by Nomura et al. (2012) reported the sensitivity and specificity of LDH to be 0.72 and 0.711, respectively, which indicates its higher diagnostic validity compared to the present study [10]. Kugahara et al. (2008) also considered ALP, LDH, and Hb as valid biomarkers for screening periodontitis in pregnant women due to their high sensitivity, specificity, and positive and negative predictive values [11].

The present findings, however, should be generalized with caution due to the small sample size, causing uncertainty. Another reason for the discrepancy between the results is the contamination of saliva with blood or other oral debris, which can distort the results. Nonetheless, we performed strict monitoring to prevent such contaminations, and the patients were asked to rinse their mouths with water for one minute before collecting the salivary samples. The lack of LDH measurements based on disease severity and absence of patients with aggressive periodontitis and gingivitis were among the main limitations of this study. Further studies with a larger sample size on different groups are suggested to obtain more conclusive results.

## 5. Conclusion

According to the present findings, salivary biomarkers, including LDH and HbA1c, cannot be used with certainty for screening chronic periodontitis, cause of low sensitivity, specificity, and positive and negative predictive values. Further studies bwithb higher sample sizes are needed to confim the results.

## Figures and Tables

**Figure 1:** Diagnostic flowchart for screening periodontal disease with level HbA1c and LDH saliva (CPI = 3) as the main cutoff is considered and DH (272), HbA1c (257) cutoff lines is calculated based on it.

**Figure 2:** ROC curve for HbA1c and LDH diagnostic value for periodontal disease assessment.

**Table 1:** Comparison of HbA1c level, LDH, PDD, and CAL based on CPI.

**CPI**	**0 (n =30)**	**3 (n =18)**	**4 (n =11)**	**P-value**
HbA1c (*μ*g/mL)	369.40 ± 172.71 (303.70 ± 435.09) CI%95	272.27 ± 86.84 (229.09 ± 315.46) CI%95	294.24 ± 121.83 (212.39 ± 376.08) CI%95	0.61
LDH IU/L	159.32 ± 206.08 (82.37 ± 236.27) CI%95	257.11 ± 319.24 (98.36 ± 415.87) CI%95	88.18 ± 83/58 (32.03 ± 144.33) CI%95	0.151
PD (mm)		2.08 ± 1.72 (2.45 ± 3.17) CI%95	2.94 ± 0.49 (2.62 ± 3.27) CI%95	0.595
CAL		2.93 ± 0.61 (2.62 ± 3.23) CI%95	4.45 ± 0.62 (4.04 ± 4.87) CI%95	<0.001

CPI, HbA1c, LDH, IU/L, PD, CAL.

**Table 2:** Comparison of HbA1c and LDH levels between patients with periodontitis and healthy individuals.

	Periodontitis		P-value
	Negative (healthy controls), n =30	Positive (patients), n =29	
**HbA1c (ug/ml)**	369.60 ± 172.71	280.60 ± 99.98	
	(303.70 ± 435.09) CI%95	(242.57 ± 318.63) CI%95	0.020
**LDH (IU/L)**	159.32 ± 206.8	193.03 ± 267.08	0.589
	(82.36 ± 236.27) CI%95	(91.44 ± 294.62) CI%95	

**Table 3:** Evaluation of the diagnostic value of salivary HbA1C and LDH levels for periodontitis screening based on the ROC curve analysis.

	**Cut-off value**	**P-value**	**Sensitivity**	**Specificity**	**Positive predictive value**	**Negative predictive value**	**AUC**
CPI	3	<0.001					
HbA1c	257	<0.001	0.64	0.27	0.51	0.27	0.385
LDH	272	<0.001	0.46	0.50	0.20	0.76	0.587

## Data Availability

No data were used to support this study.
